# Physiological Effects of Ferroptosis on Organ Fibrosis

**DOI:** 10.1155/2022/5295434

**Published:** 2022-09-30

**Authors:** Xiaojun Du, Rui Dong, Yuzhang Wu, Bing Ni

**Affiliations:** ^1^Department of Pathophysiology, Army Medical University, Chongqing 400038, China; ^2^Chongqing International Institute for Immunology, Chongqing 401338, China; ^3^Department of Immunology, Army Medical University, Chongqing 400038, China

## Abstract

Ferroptosis is a new type of programmed cell death with unique morphological, biochemical, and genetic features. From the initial study of histomorphology to the exploration of subcellular organelles and even molecular mechanisms, a net connecting ferroptosis and fibrosis is being woven and formed. Inflammation may be the bridge between both processes. In this review, we will discuss the ferroptosis theory and process and the physiological functions of ferroptosis, followed by a description of the pathological effects and the underlying mechanisms of ferroptosis in the pathogenesis of tumorigenesis, ischemic damage, degenerative lesions, autoimmune diseases, and necroinflammation. We then focus on the role of ferroptosis in the fibrosis process in the liver, lung, kidney, heart, and other organs. Although the molecular mechanism of ferroptosis has been explored extensively in the past few years, many challenges remain to be resolved to translate this information into antifibrotic practice, which is becoming a promising new direction in the field of fibrotic disease prevention and treatment.

## 1. Introduction

Fibrosis results from the maladaptive repair of tissues and organs and is a chronic and irreversible process. Almost all tissues and organs undergo fibrotic changes, particularly the liver, lungs, kidneys, and heart. In these organs, fibrosis manifests as the abnormal deposition of collagen and unbalanced extracellular matrix (ECM) homeostasis, causing irregular scar formation and distortion of the tissue structure and ultimately loss of normal function. Although fibrosis may disrupt the morphology and structure of tissues and organs, it is an orderly and delicately regulated process. In most cases, persistent damage and parenchymal cell destruction are the predisposing factors for fibrosis. Either cellular necrosis or programmed cell death (PCD) initiates the release of damage-associated molecular patterns (DAMPs), promoting sterile inflammation, immune cell activation, and the formation of local infiltrating foci [1]. Some cytokines (transforming growth factor beta (TGF-*β*), tumor necrosis factor alpha (TNF-*α*), interleukin- (IL-) 6, IL-13, and IL-33) and nonpeptidic mediators, including ROS, jointly build a proinflammatory and repair-promoting microenvironment and activate collagen-secreting mesenchymal cells, which transition from a resting state to a functional state and participate in the remodeling of the ECM to achieve tissue repair [2]. However, once parenchymal cell death persists for a long time, the damaged cells are not completely repaired and replaced by mesenchymal stem cells, and the remaining cells that are not removed from the microenvironment of the lesion lead to pathological fibrosis and scar formation and ultimately induce structural disorders and functional failure. Clearly, the modality of cell death affluences the tissue repair response and participates in key regulatory activities involved in the activation, maintenance, and outcome of fibrosis [3]. Various cell death pathways have unique physiological characteristics and different cell susceptibilities and have significant differences in regulating the fibrosis process of different organ systems.

Ferroptosis is a new type of PCD driven by lipid peroxidation that relies on the presence of abundant cellular iron. This nonapoptotic cell death mode is characterized by cystine starvation, glutathione (GSH) consumption, iron overload, and related lipid peroxidation. The aforementioned phenomenon requires a distinct GSH-dependent peroxidase, GPX4; thus, establishing the cystine/GSH/GPX4 system is considered the control center of the ferroptotic death cascade [4]. The inactivation of GPX4 is critical for the peroxidation of unsaturated fatty acids on membrane lipids, and iron ions act as an effective catalyst to promote the cell death process. Later, studies discovered some pathways independent of GPX4, including ferroptosis suppressor protein 1 (FSP1) located on the cell membrane [5, 6] and DHODH located on the inner mitochondrial membrane [7], which also modulate the signal generating ferroptosis by mediating the production of reduced ubiquinone (CoQ). In summary, the occurrence of ferroptosis is strictly regulated, and it represents a choice for cells under oxidative stress to survive or die.

Ferroptosis is an indispensable participant in many pathological processes, including cancer, ischemia-reperfusion injury, and degenerative diseases. The loss of cells and the subsequent inflammatory response are the main mechanisms in which ferroptosis plays a role, and these processes are also highly compatible with the pathogenesis of fibrotic lesions. The current results also strongly support the hypothesis that ferroptosis assumes an important role in the development of fibrotic lesions, and the underlying mechanism is not limited to tissue inflammation. In this review, we describe recent research progress in ferroptosis and focus on the mechanism of ferroptosis in fibrosis pathogenesis, including in the liver, lung, kidney, heart, and other organs. We tried to build a clear interconnected network between ferroptosis and fibrosis and to provide a novel choice for the preparation of a broad range of effective antifibrotic drugs.

## 2. Ferroptosis: A Novel Type of Iron-Dependent PCD

The balance between cell division, proliferation, and death determines the survival of multicellular organisms. During the process of evolution, multicellular organisms have continuously developed various sophisticated and procedural regulatory mechanisms to carefully maintain this balance, allowing the senescence and death of cells to occur in an orderly manner. Previously, PCD was mainly explored based on morphology. Advances in science and technology have spurred research into the molecular mechanism of cell death. We have gradually realized that a single mode of death is extremely unfavorable for cells. At the same time, pathways that differ from apoptosis, autophagy, and other classical programmed death pathways are constantly being discovered. The activation of multiple death pathways by a single stimulus has become the mainstream focus. Among these pathways, ferroptosis, a novel type of PCD, is a key link in multiple channels and plays an irreplaceable role in individual development, homeostasis, and disease.

Previous molecular targeted therapy studies have found that many clinically used anticancer drugs are more effective and active in the presence or absence of certain oncoprotein genotypes. In 2003, a study identified the new compound erastin that was selectively lethal only in cells expressing small T oncoprotein (ST) and the oncogenic allele of HRAS (RASV12). The lethal effect of erastin is mediated by a new, nonapoptotic pathway; once it occurs, cell death is rapid and irreversible [8]. In addition, in subsequent studies, another RAS-selective lethal compound, RSL3, was also shown to trigger a similar cell death phenotype, nonapoptotic, iron-dependent oxidative death [9]. In terms of cell morphology, no cell shrinkage or chromatin condensation and margination are observed during this special death process, but changes in the morphology and structure of mitochondria and enhanced lipid peroxidation have been documented [10]. The use of traditional inhibitors of apoptosis, autophagy, and pyrolysis does not inhibit the death process, but iron ion chelating agents inhibit this process [9]. In 2012, Dixon et al. first proposed the concept of “ferroptosis” to describe the peculiar cell death pathway that is inseparable from iron and lipid peroxidation [4]. In subsequent research, the potential physiological functions of ferroptosis were gradually analyzed. More cutting-edge studies have proposed that ferroptosis is also extremely active in many pathological processes, such as tumor development [11–13], neurodegenerative changes [14, 15], and fibrosis [16, 17].

### 2.1. The Classic Process of Ferroptosis

#### 2.1.1. Cystine/GSH/GPX4 System

As early as the last century, some pioneering studies have shown that cystine deprivation induces cell death, and dead cells show a unique microscopic morphology [18]. Further research found that the recovery of GSH can promote cell growth in cystine-free medium [19]. Since then, some early studies have only focused on the importance of amino acids for cell culture. However, as increasing evidence was discovered, a new cell death pathway was identified, and its principle and regulatory network gradually became clear.

GSH is known to be an irreplaceable component in the redox balance of mammalian cells. Cysteine is a rate-limiting substrate in the production of reduced GSH, which is directly taken up by neutral amino acid transporters. Under oxidative conditions, the exogenous uptake and synthesis of cysteine mainly depend on the system Xc− (cystine/glutamate antiporter), a heterodimeric amino acid transporter consisting of solute carrier family 7, member 11 (SLC7A11) and SLC3A2 linked by disulfide bonds [20]. SLC7A11 mainly controls the specific transport of cystine and glutamate, while SLC3A2 functions as a chaperone protein. SLC7A11 is the upstream initiating factor of ferroptosis. In tumor cells, inhibition of the expression and transport activity of SLC7A11 results in decreased uptake of cystine by the cell and may trigger ferroptosis of tumor cells. On the other hand, human tumor cells overexpress SLC7A11, which exhibit greater resistance to ferroptosis and weaken the effect of tumor suppressors [21]. Notably, in addition to exogenous uptake, cells also use methionine to synthesize cysteine endogenously through the transsulfuration pathway. In some cancer cells, the transsulfuration pathway is continuously activated, which is why tumor cells survive the ferroptosis storm. For example, ovarian cancer cells treated with erastin (an inhibitor of SLC7A11) for several days gradually increase the transsulfuration effect to compensate for the lack of cystine [22]. Related studies have also shown that disrupting enzymes related to the transsulfuration pathway may delay tumor growth. Therefore, these results all illustrate the indispensable role of cystine uptake in ferroptotic death.

Cystine is reduced to cysteine in cells, and GSH is synthesized through a reaction catalyzed by glutamic acid cysteine ligase (GCL) and glutathione synthase (GSS). In GPX4-mediated catalysis, GSH molecules provide electrons to reduce phospholipid peroxides to the corresponding alcohols, accompanied by the production of oxidized glutathione (GSSG) (Figure 1). When ferroptosis had not yet been defined, some researchers have established a GPX4 knockout mouse model and found that GPX4 deprivation induced the death of embryonic fibroblasts in a lipid peroxidation dependent, nonapoptotic manner; in addition, the neuron-specific loss of GPX4 leads to neurodegeneration in the mouse cortex and hippocampus [23]. After ferroptosis was identified and defined, a large amount of research data also confirmed that GPX4 is the core regulatory protein of ferroptosis and the key to cell survival. RSL3 is an inhibitor of GPX4 that induces ferroptosis by irreversibly binding to selenocysteine in the active site of the GPX4 enzyme [24]. Conversely, by upregulating the expression of GPX4, resistance to ferroptosis develops.

#### 2.1.2. Iron Metabolism

Ferroptosis is iron-dependent and lipid peroxidation-mediated cell death pathway. The Fenton reaction promotes non-enzyme-catalyzed or spontaneous lipid peroxidation. The spontaneous process is a chain reaction catalyzed by iron and oxygen, which ultimately leads to the formation of large amounts of ferroptotic marker-phospholipid hydroperoxides (PLOOHs) [25]. In addition, the catalytic activity of lipoxygenases and peroxidase requires the participation of iron. Iron is also essential for ROS production during many redox metabolism processes in cells [24]. Iron chelators or genetic inhibition of cellular iron uptake was shown to be effective in preventing ferroptosis [4].

Therefore, the uptake, utilization, storage, and export of iron all affect ferroptosis. Under normal circumstances, transferrin receptor 1 (TfR1) takes up transferrin-bound iron through receptor-mediated endocytosis and then releases the reduced Fe^2+^ into the cytoplasm. Iron ions are partially stored in ferritin, which may prevent Fe^2+^ oxidation by ROS [26]. The balance of iron intake and iron storage strictly regulates the iron ion load in cells. Suppression of transferrin or TfR1 expression significantly inhibits erastin-induced ferroptosis [9, 27]. In addition, nuclear receptor coactivator 4- (NCOA4-) mediated autophagic degradation of ferritin (ferritinophagy) is a selective form of autophagy that results in the release of Fe^2+^ and maintains the cellular labile iron contents, which are necessary for lipid peroxidation-induced ferroptosis [28, 29]. Conversely, strategies that promote the excretion of intracellular iron or inhibit the autophagic degradation of intracellular ferritin allow the cell to resist ferroptosis [28, 29](Figure 1).

#### 2.1.3. Lipid Peroxidation

Cascade-amplified lipid peroxidation is the most striking characteristic of ferroptosis. Polyunsaturated fatty acids (PUFAs) cover easily separated bis-allylic hydrogen atoms, which are susceptible to lipid peroxidation and are imperative for the implementation of ferroptosis [24]. The remodeling of the membrane lipid bilayers and the accumulation of oxidized phospholipids are certainly important drivers of ferroptosis. Through rigorous screening, acyl-CoA synthetase long-chain family member 4 (ACSL4) and lysophosphatidylcholine acyltransferase 3 (LPCAT3) are highlighted as speed-limiting components in PUFA synthesis and contribute substantially to promoting the process of ferroptosis [30, 31]. However, the current research results do not provide an answer to how membrane lipid unsaturation beyond the warning value achieves cell quenching.

In nonenzymatic lipid peroxidation, the bis-allylic hydrogen atoms from polyunsaturated fatty acyl moieties in phospholipids (PUFA-PLs) integrated into the lipid bilayer are removed by an initiating radical, which forms carbon-centered phospholipid radicals (PL•) and reacts with oxygen to create phospholipid peroxy radicals (PLOO•), which remove hydrogen from another PUFA to form PLOOH and a new PL•, triggering a series of chain reactions (Figure 1) [32, 33]. Once this automatic amplification process catalyzed by iron and oxygen loses precise control, it will cause membrane damage and cell death.

The enzymatic lipid peroxidation process is mainly executed by lipoxygenase (LOX). LOX is a nonheme iron-containing enzyme that catalyzes the dioxygenation of PUFAs to produce various PLOOH moieties [34]. However, several current studies have questioned the effect of LOX on ferroptosis. Knockout of ALOX15 does not rescue ferroptosis and its serious pathological consequences caused by GPX4 deletion [35–37]. Researchers have hypothesized that LOXs may only be involved in some cases of ferroptosis. However, the effect of enzymatic reactions on inducing ferroptosis is still unquestionable. Enzymatic reactions may produce a large amount of PLOOH, which is also necessary for ferroptosis. In addition, recent studies have also confirmed that the lack of cytochrome P450 oxidoreductase (POR) indeed significantly alleviates ferroptosis caused by GPX4 depletion [38]. The POR accidentally removes electrons from NAD(P)H to oxygen to generate H_2_O_2_, which subsequently undergoes the Fenton reaction involving iron, triggering subsequent lipid peroxidation events and thereby causing rupture of the membrane during ferroptosis [39].

### 2.2. The GPX4-Independent Ferroptotic Execution Process

#### 2.2.1. NAD(P)H/FSP1/CoQ10 System

The effect of the classic cystine/GSH/GPX4 system on regulating ferroptosis is undeniable, but the sensitivity of diverse cancer cell lines to GPX4 inhibitors is inconsistent, indicating that other regulatory signaling pathways parallel to GPX4 are involved in the process of ferroptosis. The Conrad research team at the Neuherberg Institute of Developmental Genetics in Germany assessed cells lacking GPX4 and verified FSP1 as a key factor contributing to GPX4-independent ferroptotic death [6]. Alzmann's research group at the University of California at Berkeley identified the same result at almost the same time [5]. Two studies revealed an enzyme catalytic system for the first time that offsets the absence of GPX4 during ferroptosis.

FSP1 obtains a flexible membrane binding ability through myristoylation and establishes contact with the plasma membrane, Golgi, and perinuclear structures. Mutating the myristoylation site of FSP1 causes it to lose the function of resisting ferroptosis. Further studies of the internal mechanism found that the antiferroptotic effect of FSP1 was independent of system Xc− and ACSL4 expression. Myristoylated FSP1 is recruited to the plasma membrane and participates in the reduction of CoQ10 in the presence of NADH. Reduced CoQ is an antioxidant that traps free radicals, which inhibit the spread of lipid peroxides, thereby inhibiting ferroptosis [5, 6] (Figure 1).

Later, in a study of cancer entities, pharmacological treatment with FSP1 and GPX4 inhibitors exerted a strong synergistic effect on inducing ferroptotic death. In summary, the NAD(P)H/FSP1/CoQ10 axis may be independent of and functionally parallel to the classical system, coordinating the occurrence of ferroptosis with the cystine/GSH/GPX4 axis.

#### 2.2.2. DHODH/Ubiquinol in Mitochondria

CoQ10 is mainly located on the mitochondrial and plasma membranes of mammals. Ubiquinol is the reduced form of ubiquinone (CoQ10), which has antioxidant properties. The ferroptotic death defense mechanism mediated by FSP1 is also realized through the production of ubiquinol, but the activity of FSP1 is limited to the cell membrane. These research results suggest that mitochondria may also have a similar mechanism through the production of panthenol to resist the oxidative damage of membrane lipids, thereby playing a role in regulating ferroptosis. Further research found that a key enzyme involved in the de novo synthesis of pyrimidine, human dihydroorotate dehydrogenase (DHODH), is located on the mitochondria [40]. DHODH catalyzes the conversion of dihydroorotic acid molecules into orotic acid through the oxidation of ubiquinone, thereby generating ubiquinol. DHODH repairs mitochondrial lipid oxidative damage by regenerating ubiquinol and establishes an effective system dedicated to preventing ferroptosis in mitochondria [41] (Figure 1).

Compared with the differential expression of mitochondrial-localized GPX4 in different cancer cell lines, DHODH is ubiquitously expressed. In cells with low GPX4 expression, disabling DHODH leads to the accumulation of mitochondrial lipid peroxides and the activation of ferroptotic death. In contrast, in the absence of DHODH, cells with high GPX4 expression continue to block ferroptosis [7]. DHODH and mitochondrial GPX4 act in parallel to coordinate the process of mitochondrial lipid peroxidation. GPX4, FSP1, and DHODH, which are located in designated subcellular structures, form a tripartite force to defend against ferroptosis (Figure 1).

## 3. Ferroptosis and Fibrosis

Different types of stimulation can lead to epithelial and/or endothelial injury, thus triggering complex tissue repair and wound healing procedures to restore local structure and function. After the stimulus is removed, the self-healing response will stop automatically. However, when inflammation continues or relapses, this tissue healing response will gradually amplify and become uncontrollable, initiating the irreversible fibrosis process and leading to pathological ECM formation and scarring. This fibrotic state can occur in almost every important organ and tissue of the human body. This chronic and progressive vicious cycle will eventually lead to organ degeneration. Unfortunately, an effective method to reverse the fibrosis process has not been developed. Approaches designed to delay or even reverse fibrosis have become a difficult problem that has perplexed clinicians for a long time.

Based on accumulating evidence, the occurrence of ferroptosis is always accompanied by the presence of inflammation. More interestingly, the cross-links between ferroptosis and inflammation are not unidirectional but are mutually induced and drive a local autoamplification loop [42]. The internal relationship between ferroptosis and aseptic inflammation has attracted the attention of clinical workers, and research on ferroptosis in various diseases is becoming increasingly in depth. The executive control of the occurrence and development of severe chronic diseases by ferroptosis is undeniable, and it has different responsibilities in different disease backgrounds. Intriguingly, oxidative stress, tissue damage, and aseptic inflammation cause irreversible fibrosis, changes in various organs throughout the body, and finally functional failure. Thus, an inseparable relationship must exist between ferroptosis and fibrosis. Treatments targeting ferroptosis may create new opportunities for the remedy of fibrotic diseases (Table 1).

### 3.1. Ferroptosis and Liver Fibrosis

Liver fibrosis is a common clinical pathophysiological process that is almost irreversible using existing methods. Viruses, drug toxicity, alcohol abuse, and a high-fat diet may cause chronic liver damage [43]. The injured liver maintains functional continuity and structural integrity through the regeneration and reconstruction of parenchymal cells and the formation of nonfunctional fibrous connective tissue by some mesenchymal cells. Persistent activation of hepatic stellate cells (HSCs) with a fibroblast phenotype is proposed to be responsible for the distortion and imbalance of normal liver tissue leading to fibrosis [43]. The occurrence and development of liver fibrosis correlates with pathophysiological processes such as inflammation, iron overload, and oxidative stress [44] (Figure 2). Based on these facts, liver fibrosis is likely associated with ferroptosis.

Nonalcoholic steatohepatitis (NASH) is an intermediate transition stage from simple fatty liver to cirrhosis. At present, the definite diagnosis of NASH is based not only on the deposition of fat in liver cells (steatosis) but also on the characteristic histological evidence of liver cell damage, death, inflammatory infiltration, and fibrosis [45]. Progressive fibrosis in patients with NASH has important clinical significance, but the underlying mechanism by which simple fatty liver changes to steatohepatitis and fibrosis is poorly understood. A study found that lipids induce iron efflux from hepatocytes as extracellular vesicles into neighboring HSCs, resulting in iron deficiency in hepatocytes and iron overload in HSCs. Excessive iron load directly stimulates ROS generation in HSCs, which in turn activates HSCs and promotes liver fibrosis. The aberrant distribution of iron is currently presumed to be an important link leading to hepatic steatosis and fibrosis [46]. In previous research, oxidative stress due to abnormal lipid deposition (lipotoxicity) was considered a critical upstream event in the pathogenesis of NASH. The accumulation of iron in the liver due to metabolic disorders was also believed to accelerate disease deterioration and fibrosis in individuals with NASH [47]. GPX4 expression is reduced in the liver and kidney tissues of high-fat diet-fed mice, while treatment with the ferroptosis inhibitor Fer-1 attenuates obesity-induced tissue inflammation and fibrosis [48]. Therefore, ferroptosis may play a role in the progression from inflammation to fibrosis. In a recent study, researchers used a choline-deficient, methionine-supplemented (CDE) diet to establish a model of steatohepatitis, showing that necrosis appeared earlier than apoptosis in the prophase of liver injury [49]. Moreover, necrosis inhibition did not prevent the occurrence of necrotic cell death, but the ferroptotic inhibitors Trolox and DFP almost completely protected hepatocytes from necrosis and inhibited the infiltration of immunocytes and the increase in the levels of TNF-*α*, IL-6, and other inflammatory cytokines [49]. Based on these facts, ferroptosis is probably the initial form of cell death activated in the pathogenesis of steatohepatitis. In addition, in the NASH mouse model established with a methionine-choline-deficient diet, characteristics of ferroptosis were identified, including ROS accumulation, an increased mitochondrial membrane density, and upregulation of ferroptotic death-related genes. Inhibition of ferroptosis significantly reduces liver fibrosis in mice and downregulates the expression of the fibrogenic genes TGF-*β* and collagen *α*1 [50].

Hepatocellular carcinoma (HCC) is a tumor that develops after the accumulation of metabolic and inflammatory damage over a long period. Inflammatory cell infiltration, HSC activation, and fibrotic proliferation have been recognized as powerful factors driving HCC progression [51]. Compared with normal liver tissue, ACSL4 expression was significantly upregulated in HCC tissue, suggesting that ferroptosis may be responsible for the development of HCC [52]. In most previous studies, ferroptosis has been considered an endogenous mechanism suppressing tumor growth. In contrast, a recent study found that an ACSL4-dependent process plays an unexpected cancer-promoting role in HCC formation. In an HCC model of chronic liver injury, loss of ACSL4 significantly impaired the progression of tumor growth, accompanied by lower levels of tissue fibrosis and proliferation [53]. ACSL4-dependent ferroptosis establishes a link between tissue fibrosis and tumor progression, and hepatocyte ferroptosis is a breakthrough target that aggravates fibrotic and proliferative events as a promoter of HCC growth.

Excessive iron accumulation contributes substantially to the progression of liver fibrosis and even cirrhosis, and many patients in the terminal phase have liver iron overload. The toxic effect of accumulated iron on hepatocytes is attributed to the oxidative damage caused by the Fenton reaction to produce ROS, but its role in fibrogenesis and related molecular mechanisms are unclear. According to a previous study, excessive iron completely inhibits ferroptosis in vivo and in vitro [54]. Elevated lipid peroxidation and PTGS2 mRNA expression were detected in the livers of high-iron-fed mice, accompanied by large amounts of collagen deposition and tissue fibrosis. The specific ferroptotic inhibitors Fer-1 and deferoxamine alleviated the abovementioned effects and protected against liver damage induced by iron overload [54]. Mechanistic studies revealed that a massive overdose of iron stimulated heme oxygenase-1 (HO-1) overexpression in primary hepatocytes. The continuously upregulated HO-1 causes excessive accumulation of Fe^2+^ in cells, which eventually leads to hepatocyte ferroptosis [55]. Iron overload is a necessary condition for ferroptosis, and it is also a predisposing factor for liver fibrosis. Abundant evidence has indicated that the regulation of iron homeostasis is the crossroads of ferroptotic death and fibrosis. Transferrin (Trf) is a metal-binding protein that is abundant in serum, is mainly synthesized in the liver, and correlates with the regulation of iron metabolism [56]. In a recent study, researchers specifically knocked out the Trf gene in mouse hepatocytes. In subsequent observations and evaluations, the mice exhibited iron deficiency-related anemia, tissue iron overload, and liver injury. In addition, supplying the Trf-/- mice with a high-iron diet showed that the mice were more sensitive to iron accumulation and were more susceptible to ferroptosis and liver fibrosis. However, the inhibition of ferroptosis in Trf-/- mice successfully alleviated the liver fibrosis phenotype [57]. These results illustrate the pathogenic molecular mechanism of Trf deficiency, which aggravates liver damage and liver fibrosis by inducing ferroptosis through the accumulation of non-Trf-bound iron. In subsequent studies, researchers further determined that iron accumulation in tissues and organs under Trf-deficient conditions is mediated by the metal membrane protein SLC39A14 (Zip14) [57].

The activation of HSCs is a pivotal step in the occurrence and evolution of liver fibrosis (Figure 2). Targeted interventions designed to promote the survival of HSCs represent a feasible approach for the prevention and treatment of liver fibrosis. Clinical trials of ferroptosis-inducing drugs have demonstrated that sorafenib and erastin reverse or terminate the activated phenotype of HSCs and trigger an irreversible ferroptotic cascade [58]. The expression of the RNA-binding protein ELAVL1 increased after drug treatment. Subsequent mechanistic studies found that ELAVL1 stabilizes the expression of the autophagy-related protein Beclin-1 and increases the overall level of autophagy. As the autophagic degradation of ferritin increases, HSC ferroptosis is induced [58]. Consistent studies have also proposed that sorafenib and erastin induce ubiquitination and degradation of the RNA-binding protein ZFP36, decreasing ZFP36 expression and thereby reducing the specific binding to the key autophagy gene ATG16L1 to increase the stability of the ATG16L1 mRNA and induce HSC ferroptosis in the same manner as autophagy activation [59]. Moreover, artemether promotes the expression and nuclear import of P53 and induces TP53-dependent ferroptosis of HSCs, thereby inhibiting the damage and fibrosis induced by CCl_4_ in the mouse liver [60]. In previous reports, artesunate attenuated the progression of liver fibrosis by ameliorating inflammation [61], modulating matrix metalloproteinases [62], and inducing HSC apoptosis [63]. A finding suggests that artesunate, an inducer of ferroptosis, significantly enhances ferritinophagy-mediated ferroptosis in activated HSCs, thereby ameliorating liver fibrosis. In contrast, inhibition of ferroptosis with DFO completely eliminated the artesunate-induced antifibrotic effects [64]. Magnesium isoglycyrrhizinate is a first-line anti-inflammatory and hepatoprotective agent. Mechanistic studies have shown that magnesium isoglycyrrhizinate upregulates the expression of HO-1, thereby affecting the expression of molecules downstream of HO-1 related to iron metabolism, causing intracellular iron overload and lipid peroxide accumulation to induce HSC ferroptosis and inhibit liver fibrosis [65]. Sorafenib inhibits ECM accumulation to treat liver fibrosis, which is achieved by triggering HSC ferroptosis through the inactivation of the HIF-1*α*/SLC7A11 pathway [66]. In a study of the molecular mechanism of ferroptosis in HSCs, the upregulation of the bromodomain-containing protein 7 (BRD7) protein triggers the subsequent mitochondrial translocation of P53, causing mitochondrial iron overload, enhancing respiratory chain function, and ultimately inducing ferroptosis in HSCs [67].

A review summarizes the role of ferroptosis in the pathogenesis of liver disease, which assumes different responsibilities in different disease contexts [16]. We expect to obtain more evidence at different tissue levels to construct a dynamic evolutionary process from the activation of inflammation to liver fibrosis, to cirrhosis, and eventually to hepatocellular carcinoma, enabling researchers to target the emergence or inhibition of ferroptosis at key links in the pathway. Most of the current antihepatic fibrosis drugs stop at the mechanistic level of ferroptosis. We envision future drugs that target fibrosis in a multilayered enveloping manner and enable the transition from fundamental mechanistic studies to clinical applications.

### 3.2. Ferroptosis and Lung Fibrosis

Pulmonary fibrosis is the end-stage change of a large class of lung diseases, which is defined as the formation of scars after abnormal repair of normal alveolar tissue after damage. The persistence and prolonged survival of myofibroblasts are presumed to be central events leading to excessive ECM deposition [68]. In fibrosis-related diseases such as idiopathic pulmonary fibrosis (IPF) [69, 70], bronchial asthma [71], and chronic obstructive pulmonary disease (COPD) [72], the fibroblast-to-myofibroblast transition, is one of the main mechanisms generating myofibroblasts in fibrotic lung tissue. The regulation of myofibroblasts and the occurrence of transformational events may be a shortcut to benefit patients with fibrotic lung disease. Some current studies have focused on targeting PCD of myofibroblasts to combat fibrosis, and with the in-depth analysis of the pathological effects of ferroptosis, an increasing number of studies have reported the latent capacity of ferroptosis in lung pathology (Figure 3). Some recent studies have focused on ferroptosis and pulmonary fibrosis and have obtained some results that expound on the correlation between them.

Idiopathic pulmonary fibrosis (IPF) is chronic, destructive, and irreversible and bears the hallmarks of interstitial lung disease [73]. The bronchoalveolar lavage fluid (BALF) chemistry of patients with IPF was monitored in some previous studies, and a related investigation was conducted to assess oxidative stress, lipid metabolism, and iron accumulation. These results establish a scientific theoretical foundation for the role of ferroptosis in the progression of IPF. Iron levels are significantly elevated in human lung tissue from patients with IPF, while all in vivo experiments in mice suggest a role for iron in fibrosis. At the same time, human lung fibroblasts exhibited a stronger profibrotic response upon exposure to higher iron concentrations [74]. In addition, in the study of the pathogenesis of IPF, the imbalance of redox state in lung tissue has been widely confirmed. The levels of many antioxidant proteins, including nuclear factor erythroid-2-related factor 2 (Nrf2), GSH, and GPX4, are decreased in the lung tissues from patients with IPF [75]. Interestingly, in one study, the key role of GPX4-regulated lipid peroxidation in the process of pulmonary fibrosis was highlighted. Compared with non-IPF lung fibroblasts, GPX4 levels in lung fibroblasts from patients with IPF are reduced, and enhanced lipid peroxidation associated with 4-HNE was observed [76]. Furthermore, increased lipid peroxidation due to low GPX4 expression promotes the progression of IPF by increasing the activity of the transforming growth factor beta (TGF-*β*) signaling pathway related to myofibroblast differentiation [76]. Both iron overload and lipid peroxidation regulated by GPX4 suggest the activation of ferroptosis. Therefore, these results convincingly show that ferroptosis is likely to affect the pathogenesis of IPF and the progression of fibrosis. Erastin is a classic inducer of ferroptosis and may participate in the progression of IPF by reducing GPX4 expression and promoting ROS production and lipid peroxidation. Fer1 attenuates the aforementioned effects and inhibits pulmonary fibrosis and ferroptosis [77]. In a study that screened the FerrDb database and previous studies, 19 ferroptosis-related genes (FRGs) related to the overall survival of patients with IPF were found, and a new prognostic model of IPF was established based on 5 FRGs. The model was verified to be an independent risk factor for the overall survival of patients with IPF [78]. However, the mechanisms by these genes regulate the development of IPF, and the role ferroptosis plays in IPF is unclear and worth exploring.

Radiation-induced pulmonary fibrosis (RIPF) is a late-stage complication of radiotherapy in patients with chest tumors. Patients often experience symptoms such as an irritating dry cough, shortness of breath, and chest pain, but its pathogenesis remains unclear. In previous studies, exposure to ionizing radiation (IR) was confirmed to cause continuous ROS production, which deprives unsaturated fatty acids of electrons and causes lipid peroxidation through a series of reactions [79]. This process will not only be passed to the progeny cells but might also defile nontargeted bystander cells through the communication mechanism between cells, causing extensive oxidative damage [80]. Perhaps, this extensive radioactive lung damage is directly related to IR-induced lipid peroxidation and even further ferroptosis. In the RIPF mouse model, GPX4 expression was significantly downregulated, and the ferroptosis inhibitor liproxstatin-1 antagonized this effect. More valuably, liproxstatin-1 treatment mitigated the histological changes in irradiated mice, inhibited collagen deposition, and reduced the hydroxyproline content [81]. Subsequent studies at the cellular level also suggested that liproxstatin-1 activates the Nrf2 pathway by reducing TGF-*β*1 expression, thereby attenuating profibrotic inflammatory events [81]. Therefore, ferroptosis may contribute to RIPF, and treatments suppressing ferroptosis may delay the process of fibrosis to a certain degree. Furthermore, a decrease in the level of GPX4 in lung tissue was also observed in an irradiated mouse model in another study. However, the expression of ACSL4, which promotes lipid metabolism in ferroptosis, was increased in the IR group, and lung iron deposition was also significantly increased [82] (Figure 3). Cell death is a pivotal event in RIPF. The previous results all suggest that IR directly caused the deconstruction of biological macromolecules and then initiated apoptosis, which is the major pathway mediating the decrease in the number of cells in individuals with RIPF. However, experimental results have revealed the pathological ultrastructural changes in alveolar type II (ATII) epithelial cells in radiation-exposed mice. The mitochondrial morphology of the IR group was swollen, part of the mitochondrial membrane was destroyed, and the mitochondrial cristae were blurred and disappeared [82], which are clear features of ferroptosis.

Asthma is a chronic airway inflammatory disease. Long-term and repeated inflammatory infiltration may cause organic lesions of the airway, activation, and an increase in the number of myofibroblasts in the deep subepithelial and submucosal layers, collagen deposition, and ultimately subepithelial fibrosis. This irreversible airway remodeling also causes stenosis of the airway lumen and loss of elasticity, while the epithelium is repaired [83]. Eosinophils are important inflammatory cells that infiltrate and generate foci in individuals with asthma and are very important for the progression and maintenance of chronic inflammation [84]. Previous studies have also detected higher iron levels in eosinophils [85], suggesting a greater susceptibility to ferroptosis. According to recent research results, ferroptosis inducers mediate nonclassical ferroptosis in eosinophils, thereby effectively alleviating airway inflammation and delaying the process of airway remodeling [86]. Similarly, administration of liproxstatin-1 significantly alleviated neutrophilic asthma by inhibiting bronchial epithelial cell ferroptosis, suggesting an important role for ferroptosis in disease progression and the development of airway inflammation [87].

In addition to asthma, the long-term development of many airway inflammatory diseases may lead to the occurrence of fibrotic lesions, and an increasing number of studies have shown that ferroptosis plays an important regulatory role in disease progression. Previous studies have identified iron responsive element binding protein 2 (IREB2) as a COPD susceptibility gene, and the levels of the IREB2 protein and mRNA are significantly elevated in COPD lung tissue [88]. Disruption of the iron balance and lipid peroxidation can also be observed in individuals with COPD. Researchers found that cigarette smoke induces lipid peroxidation and ferroptosis in bronchial epithelial cells through NCOA4-mediated ferritinophagy signaling. Subsequent experiments observed thicker airway walls and worsened airway inflammation in a heterozygous GPX4-deficient COPD mouse model [89]. Dihydroquercetin treatment protected against COPD by inhibiting cigarette smoke-induced ferroptosis through the Nrf2-dependent signaling pathway [90]. Inflammatory macrophage accumulation has been recognized as a key factor involved in the progression of COPD, and mechanistic studies have shown that macrophages induce increased expression of ACSL4 in AT2 cells through arachidonate-5-lipoxygenase-mediated leukotriene B4 release, thereby rendering lung epithelial cells more susceptible to ferroptosis and injury [91]. These studies suggest that ferroptosis of airway epithelial cells may be an important mechanism underlying the progression of chronic inflammation in individuals with COPD and subsequent changes in airway fibrosis. In addition, some studies have found that a mutant of *Pseudomonas aeruginosa* can promote ferroptosis in epithelial cells by increasing lipoxygenase expression to oxidize phosphatidylethanolamine. Clinical studies further show that the persistence of lower airway inflammation depends on lipoxygenase levels and activity [92]. Cystic fibrosis is a genetic disorder that often affects the respiratory system. Previous studies have documented the coexistence of the absence of GSH antioxidant defenses [93–95] and abnormalities in iron homeostasis [96–98] in the lungs from individuals with cystic fibrosis, creating favorable conditions for the occurrence of ferroptosis. Subsequent studies also confirmed that cystic fibrosis airway epithelial cells are more susceptible to ferroptosis, and the potential coexistence of necrosis and ferroptosis may be a central event in the maintenance of chronic inflammation [99]. Given these numerous facts, we must acknowledge the irreplaceable roles of ferroptosis in the persistence of inflammation and in the process of airway remodeling. Therefore, we also have a new method to control irreversible fibrotic changes in the airway.

Pulmonary fibrosis is an irreversible pathological change, and many treatment strategies are ineffective. In this process, both early activation of inflammation and subsequent cell death drive the process of fibrosis. An increasing number of studies have revealed crosstalk between ferroptosis and pulmonary fibrosis to seek treatments. Paraquat selectively accumulates in lung tissues and causes significant tissue destruction and lung fibrosis. A study reported that ferroptosis inhibitors effectively circumvent the toxicity of paraquat, and ferroptotic death may have a considerable contribution to paraquat-mediated pathological changes in lung tissue [100]. According to a recently study, dihydroquercetin has significant efficacy against silica-induced pulmonary fibrosis, ameliorating fibrotic manifestations by inhibiting ferritinophagy-mediated ferroptosis in human bronchial epithelial cells [101]. Continuous damage to ATII cells is involved in the process of lung fibrosis. Nevertheless, the mechanism regulating their death cannot be explained by conventional PCD. In previous studies, bleomycin treatment was used to construct the disease model, and obvious fibrous pathological changes were detected in the lung tissue. Further monitoring found that the iron load in the lung tissue increased, which was accompanied by the ferroptosis of ATII cells and the activation of fibroblasts [102]. Researchers have speculated that the iron metabolism disorders of ATII cells may also be related to the evolution of bleomycin-mediated pulmonary fibrosis. Subsequent research results showed that excessive iron in ATII cells catalyzed the formation of lethal lipid ROS, thereby killing ATII cells. The targeted attack of deferoxamine on ferroptosis effectively delayed or even reversed the fibrotic phenotype of lung tissue induced by bleomycin [102].

For patients with severe pulmonary fibrosis, treatment options other than lung transplantation are extremely finite, and drug therapy is disappointing and can cause serious side effects. We expect to intervene in cell fibrosis in a more precise and effective manner, and ferroptosis may be an option. An increasing number of studies are trying to analyze the effects and mechanism of ferroptosis in pulmonary fibrosis using different approaches, but many prospective targets identified in the in vitro or animal model studies have not been used in medical practice. In the future, we expect that ferroptosis will actually be used as a clinical tool to provide hope to patients with pulmonary fibrosis.

### 3.3. Ferroptosis and Renal Fibrosis

With the in-depth study of ferroptosis, extensive research indicates that ferroptosis may be the most important regulatory necrotic signaling pathway in acute kidney injury (AKI) [103]. Recurrent and severe AKI will inevitably lead to the disrupted arrangement of the kidney structure, activation of fibroblasts, and excessive accumulation of ECM, which will eventually progress to chronic kidney disease (CKD) and end-stage renal disease (ESRD). Fibrosis is inevitable in almost all ERSD cases. However, current research has not clearly clarified whether the involvement of ferroptosis places an extra fibrotic strain on the kidney.

Renal tubular epithelial cells (TECs) are the main part of the kidney that cope with various stresses and injuries. At the same time, TECs are also the cellular source of myofibroblasts [104]. In the process of renal fibrosis, TECs mediate the initial reaction after injury, and myofibroblasts serve as the final executors [105]. Unilateral ureteral obstruction (UUO) causes primary renal tubular damage due to an obstruction of urine flow, which lays a foundation for the construction of a fibrosis model [106]. By examining a UUO animal model, researchers found that mice have the pathological phenotype of renal fibrosis. In parallel, TECs also show the typical characteristics of ferroptosis. After treatment with lipoxstatin-1 to prevent ferroptosis, fibrosis and collagen production in mice were significantly reduced [105]. At the cellular level, liproxstatin-1 reduced the expression of profibrotic factors and the activation of myofibroblasts in the UUO model. Based on these experimental results, ferroptosis participates in the pathological process of renal fibrosis. In subsequent experiments, researchers used RSL3 treatment or knockdown of GPX4 in HK2 cells by RNAi to construct a cellular model of ferroptosis. HK2 cells secreted a variety of profibrotic factors during ferroptosis, which promoted the proliferation of fibroblasts and the differentiation of fibroblasts to myofibroblasts. These effects were suppressed by liproxstatin-1 [105]. In a recent study, tectorigenin treatment significantly alleviated TEC injury and fibrotic lesions in a model of UUO. Likewise, tectorigenin showed promising efficacy against erastin/RSL3-induced ferroptosis and TGF-*β*1-stimulated fibrosis in primary renal TECs. Ferroptosis inhibition with Fer-1 also alleviated TGF-*β*1-mediated tissue fibrosis [46]. Ameliorating fibrosis progression by interfering with ferroptosis in TECs may be an approach worth considering.

Generally, ferroptosis is presumed to mediate the regulated necrosis and synchronized death of functional renal TECs, which triggers the necrotic inflammatory response, leading to poor repair and fibrosis of the tissue and organ [107]. A recent study expanded the new mechanism of ferroptosis in driving persistent inflammation and irreversible fibrosis of the kidney. Researchers found that the proximal tubular (PT) cells displayed a unique proinflammatory functional status after the lesion. This PT state significantly downregulates the typical pathways defending against ferroptosis, rendering cells susceptible to ferroptosis. Even after mild injury, the genetic induction of ferroptosis is sufficient to prevent injury-related PT cells from redifferentiating into a normal state, inducing the progressive accumulation of inflammatory PT cells, generating inflammation and fibrosis signals, and promoting maladaptive repair [108] (Figure 3). The aforementioned research results illustrate that in addition to inducing the vicious feedback cycle of necrotizing inflammation, ferroptosis also promotes irreversible changes in the cell state, resulting in pathological accumulation of cells and participating in the progression of fibrosis in a non-death-inducing pathway. From the upstream initiator of the fibrosis event, it subsequently becomes the key coordinator of the cell fate for regeneration and repair. Similar processes should occur in the kidney and other organs and tissues.

Notably, 5/6 nephrectomy will lead to the excessive filtration and perfusion pressure of residual nephrons and progress to chronic interstitial fibrosis, in which iron metabolism disorders play an important role. Treatment of CKD rats with cisplatin and DFO affects the progression of renal injury and fibrosis by interfering with ferroptosis [109]. Intervention of ferroptosis by administering drugs or gene modification has become a new remedy for renal fibrosis. TECs and other cells are involved in the development of the process from kidney injury to fibrosis, and different cell death pathways also activate different signals that together modulate the process of tissue remodeling. When examining the extensive cell signaling network, establishing the connection between molecules has always been a difficult problem. However, the application of single-cell omics provides a good shortcut. A single-cell analysis has now shown that ferroptosis and pyroptosis activate inflammatory cells and promote fibrosis development in maladapted PT cells [110]. Undoubtedly, with the application of single-cell omics, more drugs and their mechanisms of interfering with ferroptosis will be discovered, which will be of great benefit to patients with CKD.

### 3.4. Ferroptosis and Myocardial Fibrosis

Myocardial fibrosis is the result of cardiac decompensation in response to various loads and the main manifestation of the progressive decline of cardiac function. Almost all heart diseases, including hypertensive heart disease, inflammatory cardiomyopathy, and metabolic cardiomyopathy, have the same outcome, myocardial fibrosis, which ultimately leads to impaired systolic and diastolic functions of the heart.

Mixed lineage kinase 3 (MLK3) is a major contributor to the process of myocardial fibrosis. In the transverse aortic constriction mouse model, MLK3 induces cardiac insufficiency and fibrosis via NF-*κ*B/NLRP3-mediated inflammation and pyrolysis in the prophase. In the advanced phase, JNK/p53-mediated oxidative stress and ferroptosis may be the main executors leading to fibrosis and heart failure [111]. Long-term hypertension potentially leads to poor myocardial remodeling and eventually heart failure. Elabela, a peptide hormone expressed in microvascular endothelial cells, was recently found to be involved in the regulation of myocardial remodeling. Administration of elabela or Fer-1 to hypertensive mice remarkably protected against angiotensin II-induced pathological myocardial remodeling. Mechanistically, elabela treatment alleviates ferroptosis in cardiac microvascular endothelial cells by regulating the IL-6/STAT3/GPX4 pathway, thereby protecting against myocardial fibrosis [112]. In addition, astragaloside IV was found to protect rats from adriamycin-induced cardiomyopathy with features of myocardial fibrosis and cardiac insufficiency [113]. The mechanistic study revealed that the antiferroptotic effect of astragaloside IV mediated by enhancing the Nrf2 signaling pathway may be part of the principle mechanism. This result also shows that adriamycin-mediated myocardial fibrosis is related to its proferroptotic activity.

In a previous study, a team of scientists in China found that heme oxygenase-1 decomposes heme in cardiomyocytes, and bound iron is dissociated and catalyzes the production of lipid peroxides to the mitochondrial membrane, causing cell ferroptosis [114] (Figure 3). Their experimental results are the first to describe the in vivo link between cardiomyocyte death and iron overload-induced ferroptosis. However, little is known about the role of ferroptosis in scar repair after myocardial injury. A quantitative proteomic analysis showed that GPX4 expression was significantly downregulated in the prophase of myocardial infarction in mice. In contrast, the expression of other GPX members of the same family was increased at the transcriptional level [115]. The specific downregulation of GPX4 indicates that GPX4 may play a role in the occurrence and development of certain pathological processes during myocardial infarction. In addition, maladaptive myocardial remodeling in obese GPX4 haploinsufficient (GPX4+/-) mice is associated with increased cardiac expression of proinflammatory and profibrotic genes [116]. In addition, iron overload or iron deficiency causes pathological changes in the myocardium, including collagen deposition and the appearance of fibrosis. Inhibition of ferroptosis induced by system Xc- aggravates angiotensin II-mediated cardiac fibrosis and dysfunction in mice, whereas Fer-1 blocks these effects [117].

Compared to other organs, the study of ferroptosis in the heart is not sufficiently mature to reveal which signaling pathways are coordinated by ferroptosis in the process of myocardial fibrosis and their potential roles. The abovementioned research results indicate that ferroptosis is indeed involved in the progression of myocardial fibrosis and is at least part of the cause of myocardial fibrosis. Treatments targeting ferroptosis to protect against myocardial remodeling should consider the particularity of cardiomyocyte physiology. The process of myocardial fibrosis involves not only chemical signals but also mechanical signals. With further research, we believe that ferroptosis is a target worth exploring.

### 3.5. Ferroptosis and Fibrosis of Other Organs

The crosstalk between ferroptosis and fibrosis has also been identified in other tissues and organs, and ferroptosis is even the core component of certain fibrosis processes. An in vivo study of salivary gland dysfunction and ferroptosis in postmenopausal animal models found that the salivary gland tissue of ovariectomized mice had typical characteristics of ferroptosis and fibrotic changes [118]. Excess lipids and iron were also detected in normal submandibular gland tissues from postmenopausal women, resulting in increased vulnerability of salivary gland cells to ferroptosis. Ferroptotic cells accelerate the pace of salivary gland dysfunction by secreting fibrogenic mediators [118]. In a model of chronic pancreatitis induced by a Lieber-DeCarli alcoholic liquid diet, pancreatic-specific GPX4 knockout mice have more significant pancreatic fibrosis than wild-type mice [119]. Ferroptotic damage can accelerate the development of chronic pancreatitis. In a study of experimental autoimmune prostatitis (EAP), ferroptosis was found to be involved in the progression of chronic prostatitis. EAP rats exhibit more pronounced interstitial fibrosis than normal rats, and inhibition of ferroptosis significantly attenuates EAP-related inflammatory cell infiltration and stromal fibrosis [120]. Local injection of rat plasma-derived exosomes (RP-Exos) into the cutaneous wounds on the backs of irradiated rats promotes ECM remodeling and collagen production. In vitro studies indicated that RP-Exos increased the expression of genes related to cell proliferation and radioresistance but downregulated the ferroptotic death pathway in irradiated fibroblasts, thereby promoting the coalescence of irradiated wounds [121]. Approaches that promote tissue repair and healing by inhibiting ferroptosis suggest that the internal connection between ferroptosis and fibrosis has broadened the diagnosis and treatment of certain diseases.

## 4. Conclusions and Perspectives

Ferroptosis is a recently identified form of PCD with characteristic changes in morphology, biochemistry, and genetics. With in-depth research, the role of ferroptosis in regulating immunity, tumor suppression, ischemia-reperfusion injury, and other pathophysiological processes has been analyzed. In the process of research, another potential role of ferroptosis has gradually attracted the attention of researchers. Many research teams were surprised to find that ferroptosis and fibrosis seem to have a specific connection that is highly consistent in many chronic diseases of organs and tissues. In different organs, research on fibrosis and ferroptosis has intensified. From the initial study of histomorphology to the exploration of subcellular organelles and even molecular mechanisms, a network connecting fibrosis and ferroptosis is being woven and formed. Inflammation and immunity may serve as the bridge between the two processes. Ferroptosis is likely an upstream triggering program that promotes the continuation of the fibrotic state by continuously stimulating the activation of the inflammatory pathway. However, the real situation is much more complicated. In some specific cases, ferroptosis may be the executor of the fibrosis process, directly causing maladaptive repair of organs and tissues.

Although innovative advances in our perspective of the molecular mechanisms of ferroptosis have been achieved in the past few years, many challenges remain to be overcome to translate the theory into clinically effective antifibrotic treatments. We look forward to the reversal of fibrosis through the regulation of ferroptosis. Translational medicine research with ferroptotic death as the target will become a promising new direction in the field of fibrotic disease prevention and treatment.

## Figures and Tables

**Figure 1:** Three defense mechanisms of ferroptosis. Iron-catalyzed phospholipid peroxidation is the ultimate executor of ferroptosis, resulting in the accumulation of large amounts of peroxides and rupture of the cell membrane. In addition, cells immediately die. In the violent ferroptotic process, at least three cellular antioxidant systems coordinate the redox balance and defend against ferroptosis. The cystine/GSH/GPX4 system located in the cytoplasm and mitochondria is the most classic and well-studied antiferroptotic mechanism. GPX4 adapts its catalytic activity to circumvent the toxicity of lipid peroxide and maintain the stability of the membrane lipid bilayer. In addition, the cytoplasmic NAD(P)H/FSP1/CoQ10 system and mitochondrial DHODH/ubiquinol (CoQH2) system play a protective role independent of GPX4, producing CoQH2 in different subcellular locations, neutralizing lipid peroxidation, and resisting ferroptosis. System Xc-: cystine/glutamate antiporter; GSR: glutathione reductase; GSSG: glutathione (oxidized); GPX4: glutathione peroxidase 4; NCOA4: nuclear receptor coactivator 4; ACSL4: acyl-CoA synthetase long-chain family member 4; LPCAT3: lysophosphatidylcholine acyltransferase 3; PUFA: polyunsaturated fatty acid; PLOOH: phospholipid hydroperoxide; FSP1: ferroptosis suppressor protein 1; DHODH: dihydroorotate dehydrogenase; FMN: flavin mononucleotide; FMNH2: flavin mononucleotide (reduced); CoQ: ubiquinone; CoQH2: ubiquinol; SLC7A11: solute carrier family 7, member 11; SLC3A2: solute carrier family 3, member 2.

**Figure 2:** Ferroptosis and liver fibrosis. The liver is the organ most vulnerable to fibrosis. Sustained activation of inflammation and a high-iron load have been confirmed to be high-risk factors for liver fibrosis in the previous studies, and recent results have confirmed the contribution of ferroptosis to the progression of fibrosis. Ferroptosis is the linchpin at the intersection of inflammation and iron overload. It is the main death pathway activated in hepatocytes in the early stage of fibrosis. The factors exacerbating the iron load include the upregulation of transferrin and NTBI ion channel (SLC39A14) under the condition of low transferrin levels, which will accelerate fibrosis through the induction of ferroptosis. However, in HSCs, the induction of ferroptosis of activated HSCs by regulating ferritinophagy inhibits the progression of fibrosis. TfR1: transferrin receptor 1; HO-1: heme oxygenase-1; HSC: hepatic stellate cell; SLC39A14: solute carrier family 39 (zinc transporter), member 14.

**Figure 3:** Ferroptosis in the lung, heart, and kidney. In various organs and tissues, lipid peroxidation, necroinflammation, and iron overload will cause the destruction of parenchymal cells, which will lead to pathological fibrous accumulation and expedite the process of tissue and organ fibrosis. Ferroptosis seems to be intimately involved in reducing the cell number and may even be the main executor. Therefore, an oxidation imbalance, inflammation, and the iron load form a bridge between ferroptosis and fibrosis. However, in different tissues and organs, the interaction between ferroptosis and fibrosis has different manifestations. (Lung) Continuous or intermittent irradiation with ionizing radiation may cause extensive pulmonary fibrosis. This extensive injury is related to lipid peroxidation caused by ionizing radiation and ferroptosis mediated by multiple pressures. (Heart) The activation of HMOX1 mediated by Nrf2 signaling leads to the dissociation of iron ions from heme, excessive accumulation in cardiomyocyte mitochondria, and the activation of ferroptosis, resulting in myocardial injury and subsequent fibrosis. (Kidney) Proximal tubule cells form a special proinflammatory state after injury, rendering them more vulnerable to ferroptosis. In this special environment, even if the injury is lower than the defense threshold, the induction of ferroptosis might also affect the normal repair of cells and eventually induce fibrosis. TGF-*β*: transforming growth factor; ACSL4: acyl-CoA synthetase long-chain family member 4; Nrf2: nuclear factor erythroid-2-related factor 2; ARE: antioxidant response element; HMOX1: heme oxygenase-1; PTCs: proximal tubule cells.

**Table 1:** The role of ferroptosis in fibrosis.

Organ	Mechanism	Molecular foundation	Ref
Liver	Iron overload-induced toxicity	Iron distribution disorder: iron in hepatocytes is excreted into adjacent HSCs through extracellular vesicles.	[46]
		Iron overload promotes ferroptosis in hepatocytes by inducing HO-1 overexpression.	[55]
		Trf-TFR1 mediates iron accumulation and causes ferroptosis in hepatocytes.	[57]
		Zip14-mediated accumulation of NTBI causes ferroptosis in hepatocytes with a Trf deficiency.	[57]
	Hepatic stellate cell activation	The RNA-binding protein ELAVL1/HuR induces HSC ferroptosis by regulating the autophagy pathway.	[58]
		The RNA-binding protein ZFP36/TTP protects against ferroptosis by regulating the autophagy signaling pathway in HSCs.	[86]
		Artemether ameliorates liver fibrosis by inhibiting HSC activation via p53-dependent ferroptosis.	[60]
		Artesunate ameliorates hepatic fibrosis by mediating HSC ferritinophagy.	[64]
		Magnesium isoglycyrrhizinate ameliorates hepatic fibrosis by inhibiting HSC activation via HO-1-mediated ferroptosis.	[65]
		Sorafenib attenuates liver fibrosis by triggering hepatic stellate cell ferroptosis via the HIF-1*α*/SLC7A11 pathway.	[120]
		Wogonoside alleviates liver fibrosis by inducing SOCS1/P53/SLC7A11-mediated HSC ferroptosis.	[122]
		The BRD7-P53-SLC25A28 axis plays an important role in the ferroptosis of HSCs.	[67]
	Activation of inflammation	Ferroptotic cells release DAMPs to exacerbate tissue inflammation and fibrosis.	[44]
Lung	Fibroblast-to-myofibroblast differentiation	GPX4 inhibits and upregulates TGF-*β* signaling to promote pulmonary fibrosis.	[76]
		Erastin promotes fibroblast-to-myofibroblast differentiation by increasing lipid peroxidation and inhibiting GPX4 expression.	[77]
	Oxidative damage	Liproxstatin-1 activates the Nrf2 pathway by weakening TGF-*β* expression to attenuate RILF.	[81]
		DHQ exerts antifibrotic effects by inhibiting ferroptosis through the downregulation of LC3 and upregulation of FTH1 and NCOA4 in activated HBE cells.	[101]
	Activation of inflammation	Accumulating inflammatory macrophages induce AT2 cell ferroptosis via the ALOX5-LTB4-ACSL4 axis.	[91]
Kidney	Activation of inflammation	Ferroptotic cells release profibrotic factors (TGF-*β*, CTGF, and PDGF).	[105]
		Accumulation of proinflammatory PT cells significantly downregulates GSH to increase inflammation and fibrosis.	[106]
		Tectorigenin alleviates fibrosis by inhibiting ferroptosis in TECs through the Smad3-NOX4 pathway.	[46]
Heart	Oxidative damage	MLK3-JNK/p53 pathway-mediated oxidative stress and ferroptosis cause myocardial fibrosis.	[111]
		Astragaloside IV inhibits adriamycin-induced cardiac ferroptosis by enhancing Nrf2 signaling.	[113]
		Elabela antagonizes ferroptosis by regulating the IL-6/STAT3/GPX4 signaling pathway to prevent adverse myocardial remodeling.	[112]
Submandibular gland	Activation of inflammation	Ferroptotic cells accelerate salivary gland fibrosis by secreting IL-1 and TNF-*α*.	[118]
